The article "Effects of Perinatal Cognitive Behavioral Therapy on Delivery Mode, Fetal Outcome, and Postpartum Depression and Anxiety in Women" was published in 2022. Journal: Comput Math Methods Med.

# Effects of Perinatal Cognitive Behavioral Therapy on Delivery Mode, Fetal Outcome, and Postpartum Depression and Anxiety in Women

**DOI:** 10.1155/2022/8304405

**Published:** 2022-09-26

**Authors:** Xiuqin Guo, Xiuling Guo, Ruijun Wang, Yuan Zhang

**Affiliations:** ^1^College of Humanities Education, Inner Mongolia Medical University, Hohhot, Inner Mongolia 010059, China; ^2^Obstetrics and Gynecology Department, The Affiliated Hospital of Inner Mongolia Medical University, Hohhot, Inner Mongolia 010059, China; ^3^School of Health Management, Inner Mongolia Medical University, Hohhot, Inner Mongolia 010110, China

## Abstract

**Objective:**

To explore the effects of perinatal cognitive-behavioral therapy on delivery mode, fetal outcome, and postpartum depression and anxiety in women.

**Methods:**

The clinical data of 88 perinatal pregnant women who came to our hospital from May 2020 to May 2021 were retrospectively analyzed and grouped into the routine group and the cognitive behavioral intervention group according to different perinatal nursing methods, with 44 cases in the cognitive behavioral intervention group received by cognitive behavioral therapy, and 44 cases in the routine group obtained by routine obstetric care during the perinatal period. The anxiety of pregnant women was evaluated by the Hamilton Anxiety Scale (HAMA). The positive cooperation and negative response of the perinatal pregnant women in two groups were recorded. The trial delivery rate, mode of delivery, amount of intrapartum bleeding, neonatal Apgar score, and visual pain simulation score (VAS) within 48 hours after delivery of the pregnant women in the two groups were also recorded and compared. The incidence of depression of pregnant and lying-in women in the two groups was recorded on the 5th and 42nd day after delivery.

**Results:**

After the intervention, the anxiety score of pregnant women in the cognitive behavioral intervention group was significantly lower than that in the routine group (*P* < 0.05). Following the intervention, the positive cooperation score of pregnant women in the cognitive behavioral intervention group was prominently higher than that in the routine group, and the negative cooperation score was observably lower than that in the routine group (*P* < 0.05). The rate of spontaneous delivery in the cognitive behavioral intervention group was significantly higher than that in the conventional group (*P* < 0.05), while the VAS score and blood loss in the cognitive behavioral intervention group were notably lower than those in the routine group (*P* < 0.05). The proportion of women with EPDS score <9 points, i.e., no postpartum depression both on the 5th and 42nd day after delivery, were significantly higher than those in the routine group (*P* < 0.05), whereas the proportion of patients with postpartum depression symptoms scored 9–13 points were markedly lower than those of the routine group (*P* < 0.05).

**Conclusion:**

The cognitive behavioral therapy can improve the adverse physiological and psychological reactions of pregnant women with perinatal anxiety disorder, enhance the natural delivery rate and postoperative recovery, reduce the risk of neonatal asphyxia, and ensure the safety of mothers and infants in the perinatal period. Compared with routine nursing, this intervention method is more targeted and scientific, and is worthy of clinical promotion.

## 1. Introduction

The period from 28 weeks of pregnancy to one week after delivery is called the perinatal period. As the delivery period gets closer and closer, pregnant women will have a series of physiological and psychological reactions, which are physiologically accompanied by the changes of related hormone levels and the reduction of immune function. Psychologically, pregnant women worry too much about the fetus and the outcome of delivery as the delivery period approaches, resulting in tension, anxiety, and other adverse emotions. The adverse state may lead to endocrine mechanism disorders, and further affects multiple organ functions. In recent years, the anxiety and depression of pregnant and lying-in woman in China are increasing day by day. It has been shown that prenatal anxiety and depression increase the rate of cesarean section, lead to prolonged labor, increase the risk of postpartum hemorrhage, and even affect the development of fetal brain [1]. Therefore, it is of great significance to understand the psychological status of pregnant women and formulate relevant intervention measures for maternal and infant outcomes.

Cognitive behavioral therapy is a combination of both cognition and behavior, during which the process of cognition determines the influence of behavior, and the change of behavior can also change cognition [2]. Based on the theory of human cognitive process, cognitive behavioral therapy changes bad cognition by changing thinking, belief, and behavior, thus solving a series of physiological and psychological problems of patients. At present, cognitive behavioral therapy has been widely used in the treatment of psychological diseases [3, 4]. Some scholars have conducted a comparative study on cognitive behavioral therapy for patients with generalized anxiety disorder, and found that cognitive behavioral therapy is conducive to controlling and ameliorating anxiety disorder, improving patients' negative emotions, and the quality of life [5, 6].

This study mainly analyzed the efficacy of cognitive behavioral therapy in the treatment of perinatal anxiety symptoms, which could provide evidence-based medical proof for the clinical application of cognitive behavioral therapy.

## 2. Materials and Methods

### 2.1. General Materials

This study was approved by the Ethics Committee of our hospital. A total of 88 pregnant women with perinatal anxiety disorder who came to our hospital from May 2020 to May 2021 were selected as the research objects. The inclusion criteria are as follows: (1) all pregnant women met the diagnosis of anxiety disorder according to the mental disorder classification and diagnosis table [7], with Hamilton Anxiety Rating Scale (HAMA) [8] of ≥14 points; (2) pregnant women with no other pathological changes of body organs; (3) pregnant women were able to understand and complete the contents of the treatment without language communication barriers; (4) the pregnant women and their families agreed and signed after comprehending the study; (5) pregnant women at or above 28 weeks of gestation; and (6) first-time mothers with no history of depression at the time of enrollment. The exclusion criteria are as follows: (1) pregnant women with severe pregnancy reaction; (2) pregnant women with serious pregnancy complications and ectopic pregnancy; (3) pregnant women at less than 37 weeks of gestation; (4) pregnant women with mental disease and central nervous system disease; and (5) pregnant women who were not willing to participate in the project or could not adhere to regular postpartum follow-up. According to different perinatal nursing methods, 44 cases in the cognitive behavioral intervention group were received by cognitive behavioral therapy, while 44 cases in the routine group were obtained by routine obstetric care during the perinatal period. In the cognitive behavioral intervention group, the age of participants was between 22 and 35 years old with the average of 28.65 ± 3.91 years old, and the gestational weeks ranged from 28 weeks to one week after delivery with the average of 37.04 ± 2.25 weeks. In the routine group, the age of participants was between 22 and 37 years old with the average of 29.19 ± 4.26 years old, and the gestational weeks ranged from 29 weeks to one week after delivery with the average of 37.56 ± 3.87 weeks. No significant differences existed in age and gestational age between the two groups (*P* > 0.05). The process of general data selection is exhibited in Figure 1.

### 2.2. Methods

The participators in the routine group received routine obstetric nursing. According to the traditional nursing experience, we should have an intervention with the pregnant women, including explaining the delivery process, mechanism, and precautions to the pregnant women. To solve the delivery problems raised by the pregnant women, we need to record the sleep status of the pregnant women, conduct psychological counseling, and complete the corresponding psychological questionnaire.

The participators in the cognitive behavioral intervention group received cognitive behavioral therapy on the basis of the interventions as the routine group. Before nursing, an in-depth communication with pregnant and lying-in women was conducted, each pregnant and lying-in woman's cognition and existing adverse emotions were evaluated, the real psychological characteristics of pregnant women were understood, and their existing adverse thinking was supported and understood, thus providing a basis for formulating cognitive behavioral intervention plans. The specific steps were as follows.

1. Cognitive remodeling: the face-to-face communication was done with pregnant women to understand their most concerned problems and the causes of anxiety, with full affirmation of the positive sexual behavior of pregnant women, and the negative behavior and cognition of pregnant women were corrected. Some mothers exaggerated the risks of pregnancy complications and childbirth complications, and caused fear and anxiety due to excessive worry. Health education knowledge manuals, slide shows and other easy-to-accept formats should be used to help pregnant women establish correct cognition and guide pregnant women to vent their emotions and encourage them to talk, so as to reduce the uncertainty and anxiety level of pregnant women. In addition, the nursing staff should explain a series of physiological changes in the body once childbirth begins, and describe the hazards of negative emotions, such as affecting the function of the body's air supply, resulting in the inability of immune mechanisms to fully exert their effects, and increasing the risk of postpartum hemorrhage. The nursing staff should also instruct pregnant women how to self-regulate their emotions, and at the same time mobilize the maternal social support system to give full play to its support role in the stress state of childbirth, so as to improve the safety of childbirth
2. Behavior training: a one-on-one approach was used, including attention shifting, music therapy, and progressive muscle relaxation. During training, the room should be quiet. Attention shifting method: to guide pregnant women to divert their attention through chatting, watching dramas, and other recreational activities in case of anxiety, depression, and other adverse situations, so as to achieve the purpose of alleviating anxiety. Music therapy: to guide pregnant women to play some relaxing and soothing music in case of anxiety, depression and other adverse emotions. During this process, pregnant women could be instructed to master the correct breathing method. They could sit or stand, breathe deeply to make the air reach the lungs, and then slowly exhale the gas with 10 times repetition for 5 minutes each time to relieve tension and fear, so that the pregnant and lying-in women could relax and breathe correctly after they enter the labor process.
3. Progressive muscle relaxation: the relaxation training could be conducted using the portable skin temperature biofeedback instrument combined with progressive muscle relaxation guidance recording. The contraction and relaxation of head, neck, shoulder, chest, hands, abdomen, lower limbs, and feet were completed in the order of voice prompts, 30 minutes each time, once in the morning and once in the evening every day.

### 2.3. Outcome Measures

1. The trained therapist distributed the questionnaire to the pregnant women and introduced the precautions when filling in the form, so as to ensure that the pregnant women could check their actual situation in the recent week after understanding the meaning of each item. After the survey was completed, the general data of all pregnant women could be collected, including the age, gestational week, education background, permanent residence, life satisfaction, abortion history, pregnancy preparation, gender expectation, payment method, childbirth preparation, expected childbirth method, and postpartum care
2. The anxiety of pregnant and lying-in women was evaluated according to the HAMA scale which consisted of 2 items. Each item included 7 factors, a total of 14 factors. Each factor adopted the 5-level scoring method of 0~4 points, that was, 0 points for asymptomatic cases, 1 point for mild degree, 2 points for moderate, 3 points for severity, and 4 points for extreme weight. A score of ≥14 points was judged as mild anxiety, and a score of ≥29 points was judged as severe anxiety
3. Before the intervention, the positive cooperation and negative response of the pregnant women in the two groups were recorded, and the cooperation of pregnant women in two groups after the intervention was compared. According to the investigation regulations, the score of “not using” intervention measures was 0, the score of “occasionally using” was 1, the score of “sometimes using” was 2, and the score of “often using” was 3. The total score of 0~32 points was positive cooperation with the investigation, and 0~26 points were a negative response
4. Clinical data indicators including the rate of production trial from vagina, delivery mode, amount of intrapartum hemorrhage, neonatal Apgar score, and the score of maternal pain within 48 hours after delivery assessed using Visual analog scale (VAS) in the two groups were collected
5. Evaluation of postpartum depression: 88 pregnant and lying-in women were followed up to 42 days postpartum. The Edinburgh Postpartum Depression Scale (EPDS) with a full score of the scale of 30 points [9] was used to evaluate maternal depression at 5 days postpartum and 42 days postpartum, respectively. A score of <9 points indicated postpartum depression, a score of 9–13 points indicated postpartum depression symptoms, and a score of ≥13 points indicated postpartum depression

### 2.4. Statistical Analysis

The data were analyzed using SPSS 22.0 statistical software. The measurement data were expressed in (^−^*x* ± *s*), and the enumeration data were expressed in (%). The comparison of normally distributed measurement data between the two groups was performed by independent samples *t* test, and the comparison before and after intervention was performed by paired *t* test. Wilcoxon rank sum test was used to compare the differences of measurement data that did not conform to the normal distribution. Enumeration data were analyzed using the *χ*^2^ test or Fisher's exact test (two-tailed). *P* < 0.05 meant that the difference was statistically significant.

## 3. Results

### 3.1. Comparison of Clinical Data between the Two Groups

No significant differences existed in general data between the cognitive behavioral intervention group and the routine group (*P* > 0.05) (Table 1).

### 3.2. Comparison of Anxiety Scores between the Two Groups before and after Intervention

Before the intervention, there was no significant difference in perinatal anxiety scores between the two groups (*P* > 0.05). After the intervention, the pregnant women in the cognitive behavioral intervention group had lower anxiety scores than the women in the routine group (*P* < 0.05) (Table 2).

### 3.3. Comparison of Coordination Degree between the Two Groups before and after Intervention

No significant differences were observed in the scores of positive cooperation and negative cooperation between the two groups before intervention (*P* > 0.05). After the intervention, the pregnant women in the cognitive behavioral intervention group had a higher score of positive cooperation and a lower score of negative cooperation than the women in the routine group (both *P* < 0.05) (Table 3).

### 3.4. Comparison of Delivery Modes between the Two Groups

After the cognitive behavioral therapy intervention, the mode of delivery of pregnant women in the two groups was compared. The women in the cognitive behavioral intervention group had a higher spontaneous delivery rate than the women in the routine group (*P* < 0.05) (Table 4).

### 3.5. Comparison of Apgar Scores of Newborns between the Two Groups

After the intervention, Apgar scores of newborns in the two groups were compared. The results showed that the cognitive behavioral intervention group had a much higher proportion of newborns with Apgar scores of 8~10 than those in the routine group (*P* < 0.05) (Table 5).

### 3.6. Comparison of Intraoperative Bleeding Volume and Pain Score between the Two Groups

VAS and bleeding volume during delivery were compared between natural parturient in the two groups. The women in the cognitive behavioral intervention group had lower VAS score and bleeding volume than the women in the routine group (*P* < 0.05) (Table 6).

### 3.7. The Incidence of Depression in the Two Groups on the 5th Day after Delivery

The proportion of women with EPDS score of <9 points, i.e., no postpartum depression on the 5th day after delivery, were significantly higher than that in the routine group (*P* < 0.05), whereas the proportion of patients with postpartum depression symptoms who scored 9–13 points were markedly lower than those of the routine group (*P* < 0.05) (Table 7).

### 3.8. The Incidence of Depression in the Two Groups on the 42nd Day after Delivery

The proportion of women with EPDS score of <9 points on the 5th day after delivery were significantly higher than those in the routine group (*P* < 0.05), while the proportion of patients with EPDS score of 9–13 points were markedly lower than those of the routine group (*P* < 0.05) (Table 8).

## 4. Discussion

The perinatal period is the period from the 28th week of pregnancy to the first week of postpartum, which is a very important period before and after delivery. With the obviously increasing frequency of perinatal anxiety in pregnant women, more and more attention is paid to perinatal anxiety [10, 11]. Mood swings during pregnancy can lead to insomnia in pregnant women. Lack of sleep not only affects maternal physiological function but also leads to fetal growth retardation and even fetal deformity. Pain during childbirth is a key stressor, which can easily lead to increased cesarean section or midwifery rate, induce postpartum hemorrhage, and affect postpartum lactation. Studies have shown that the anxiety of a cesarean section is higher than that of vaginal delivery. Lack of sleep and high psychological pressure are more likely to lead to premature birth [12]. Foreign studies indicate that the incidence of antenatal anxiety is between 5.0% and 16.5%, and is still gradually increasing in recent years. Systematic and scientific perinatal nursing intervention is of great significance to promote the emotional stability of pregnant women. Therefore, it is essential to implement the necessary cognitive behavioral intervention for pregnant women with anxiety disorder.

Cognitive behavioral therapy changes people's cognition from psychological, physiological, and spiritual levels by changing people's thoughts and beliefs, so as to eliminate people's negative emotions and behaviors [14, 15]. Cognitive behavioral therapy is based on positive psychology. Clinical studies have confirmed that cognitive behavioral therapy can fully ease the anxious state of hemodialysis patients, cancer patients, and patients with generalized anxiety disorder, enhance their self-confidence, and improve treatment compliance and quality of life [16]. Cognitive behavioral therapy application helps pregnant women get rid of negative emotions in the perinatal period. The medical staffs gradually help the pregnant women correct the wrong understanding during the long-term treatment process by communicating step-by-step. Thus, the pregnant women can recognize their current problems and establish a new understanding. At the same time, pregnant women should be given timely encouragement to help them rebuild confidence and broad cognitive concepts [17]. Relevant foreign studies point out that cognitive behavioral nursing intervention improves maternal immune mechanism and enhances maternal and infant immunity by alleviating anxiety and tension [18]. The present study showed that the pregnant women in the cognitive behavioral intervention group had a much lower anxiety score than the women in the routine group after the intervention, indicating that cognitive behavior intervention therapy could alleviate the anxiety of pregnant women. The reason might be that cognitive behavioral therapy helped the pregnant women fully understood the delivery knowledge and delivery complications during the perinatal period. At the same time, targeted strategies for eliminating the negative thinking of the pregnant women were conducted to make them master emotion regulation method and improve the quality of delivery.

The present study showed that the pregnant women in the cognitive behavioral intervention group had a higher score of positive cooperation and a lower score of negative cooperation than the women in the routine group after the intervention. It can be seen that cognitive behavioral therapy has greatly mobilized the enthusiasm of pregnant women to actively participate in the delivery process and actively deal with the delivery pain and uncertain delivery outcome. Some scholars have found that cognitive behavioral therapy can not only ease maternal anxiety and depression, but also improve the rate of spontaneous delivery and breast-feeding and reduce the incidence of neonatal asphyxia during delivery [19]. The results of this study showed that the participants in the cognitive behavioral intervention group had a much higher natural spontaneous labor rate and proportion of neonatal Apgar scores of 8~10 than the routine group, suggesting that cognitive behavioral therapy could improve the rate of spontaneous labor and reduce the risk of neonatal asphyxia. The reason may be that cognitive behavioral therapy not only lay emphasis on the health education of maternal delivery knowledge but also emphasize the benefits of delivery mode on breast milk and postpartum, which could both promote the health of newborns [20]. This present study also showed that women in the cognitive behavioral intervention group had much lower VAS score and bleeding volume than in the routine group. It may be that the cerebral cortex is suppressed by anxiety, resulting in reduced oxytocin secretion, weakening uterine contraction, and increased bleeding during delivery [21]. The results of this study also showed that the proportion of patients without postpartum depression at 5 and 42 days postpartum in the cognitive behavioral intervention group were significantly higher than those in the routine group, and the proportion of pregnant women diagnosed with depression at 42 days postpartum were significantly lower than that in the routine group, further illustrating that cognitive behavioral therapy can reduce the incidence of postpartum depression while improving maternal prenatal anxiety.

In conclusion, cognitive behavioral therapy can improve the adverse physiological and psychological reactions of pregnant and lying-in women with perinatal anxiety disorder, improve the natural delivery rate and postoperative recovery, reduce the risk of neonatal asphyxia, ensure the safety of mothers and infants in the perinatal period, and be consistent with routine nursing. In comparison with routine nursing, this intervention method is more targeted and scientific, and is worthy of clinical promotion. In this study, the prenatal anxiety status of pregnant women was screened according to the definition of the perinatal period, but the pregnancy period was divided into early, middle, and late pregnancy. Therefore, the anxiety status of the whole prenatal period in this study does not represent the anxiety status of pregnant women in rectifying the prenatal period. A large sample, multicenter, long-term follow-up study is needed throughout pregnancy.

## Figures and Tables

**Figure 1:** Process of general data selection.

**Table 1:** Comparison of clinical data between the two groups [*n* (%)].

General data	Classification	The cognitive behavioral intervention group (*n* = 44)	The routine group (*n* = 44)	*χ* ^2^	*P*
Age (years)	<30	15 (34.09)	16 (36.37)	0.054	0.974
	30~40	24 (54.55)	23 (52.27)		
	>40	5 (11.36)	5 (11.36)		
Gestational week (weeks)	28~33	9 (20.45)	10 (22.73)	0.322	0.852
	34~42	26 (59.10)	27 (61.36)		
	One week after delivery	9 (20.45)	7 (15.91)		
Education background	Junior high school and below	5 (11.36)	6 (13.64)	0.558	0.906
	High school and technical secondary school	12 (27.27)	14 (31.82)		
	College and undergraduate	19 (43.18)	18 (40.91)		
	Graduate and above	8 (18.18)	6(13.64)		
Permanent residence	City	22 (50.00)	21 (47.73)	0.232	0.890
	Town	16 (36.36)	18 (40.91)		
	Village	6 (13.64)	5 (11.36)		
Life satisfaction	Satisfaction	25 (56.82)	26 (59.09)		0.863
	Ordinary	16 (36.36)	14 (31.82)		
	Dissatisfaction	3 (6.82)	4 (9.09)		
Abortion history	0	28 (63.64)	25 (56.82)		0.548
	1~2	15 (34.09)	16 (36.36)		
	≥3	1 (2.27)	3 (6.82)		
Pregnancy preparation	Sufficient	19 (43.18)	18 (40.91)	0.050	0.975
	General	21 (47.73)	22 (50.00)		
	Not ready	4 (9.09)	4 (9.09)		
Gender expectation,	Boy	8 (18.18)	9 (20.45)	0.076	0.963
	Girl	6 (13.64)	6 (13.64)		
	All can be	30 (68.18)	29 (65.91)		
Payment method	At his own expense	24 (54.55)	25 (56.82)	0.046	0.830
	Medical insurance	20 (45.46)	19 (43.18)		
Childbirth preparation	Sufficient	12 (27.27)	13 (29.55)	1.863	0.393
	General	28 (63.64)	23 (52.27)		
	Not ready	4 (9.09)	8 (18.18)		
Expected childbirth method	Spontaneous labor	38 (86.36)	33 (75.00)	1.823	0.177
	Cesarean section	6 (13.64)	11 (25.00)		
Postpartum care	Husband's family	24 (54.55)	25 (56.81)		0.844
	Mother's family	18 (40.91)	16 (36.36)		
	Maternity matron	2 (4.55)	3 (6.82)		

**Table 2:** Comparison of anxiety scores between the two groups before and after intervention ($\overset{-}{x}\pm s$).

Groups	Before intervention	After intervention	*t*	*P*
The cognitive behavioral intervention group (*n* = 44)	22.35 ± 4.51	10.42 ± 2.38	15.518	<0.001
The routine group (*n* = 44)	23.74 ± 2.25	18.14 ± 4.13	7.898	<0.001
*t*	1.829	10.743		
*P*	0.071	<0.001		

**Table 3:** Comparison of coordination degree between the two groups before and after intervention ($\overset{-}{x}\pm s$).

Groups	Positive cooperation (score)		Negative cooperation (score)	
	Before Intervention	After Intervention	Before Intervention	After Intervention
The cognitive behavioral intervention group (*n* = 44)	2.11 ± 0.52	2.32 ± 0.47	2.21 ± 0.48	1.98 ± 0.37
The routine group (*n* = 44)	2.13 ± 0.51	1.98 ± 0.62	2.18 ± 0.53	2.25 ± 0.48
*t*	0.182	2.899	0.278	2.955
*P*	0.856	0.004	0.781	0.004

**Table 4:** Comparison of delivery modes between the two groups [*n* (%)].

Groups	Delivery modes		
	Spontaneous labor	Cesarean section group due to medical factors	Cesarean section group due to nonmedical factors
The cognitive behavioral intervention group (n = 44)	31 (70.45)	8 (18.18)	5 (11.36)
The routine group (n = 44)	23 (59.09)	6 (13.64)	15 (34.09)
*χ* ^2^	6.471		
*P*	0.039		

**Table 5:** Comparison of Apgar scores of newborns between the two groups [*n* (%)].

Groups	Scores of 0~3	Scores of 4~7	Scores of 8~10
The cognitive behavioral intervention group (*n* = 44)	0 (0.00)	2 (9.09)	42 (90.91)
The routine group (*n* = 44)	0 (0.00)	8 (18.18)	36 (81.82)
*χ* ^2^	4.062		
*P*	0.044		

**Table 6:** Comparison of intraoperative bleeding volume and pain score between the two groups ($\overset{-}{x}\pm s$).

Groups	VAS (score)	Bleeding volume (mL)
The cognitive behavioral intervention group (31 cases of spontaneous labor)	5.56 ± 2.13	200.36 ± 54.21
The routine group (23 cases of spontaneous labor)	8.19 ± 1.89	289.91 ± 50.18
*t*	11.468	3.551
*P*	<0.001	0.001

**Table 7:** The incidence of depression in the two groups on the 5th day after delivery [*n* (%)].

Groups	Cases	<9	9~13	≥13
The cognitive behavioral intervention group	44	38 (86.36)	6 (13.64)	0 (0.00)
The routine group	44	29 (65.91)	14 (31.82)	1 (2.27)
*χ* ^2^		5.066	4.141	1.012
*P*		0.024	0.042	0.315

**Table 8:** The incidence of depression in the two groups on the 42nd day after delivery [*n* (%)].

Groups	Cases	<9	9~13	≥13
The cognitive behavioral intervention group	44	36 (81.82)	7 (15.91)	1 (2.27)
The routine group	44	23 (52.27)	13 (29.55)	8 (18.18)
*χ* ^2^		8.692	2.329	6.065
*P*		0.003	0.127	0.014

## Data Availability

All data, models, and code generated or used during the study appear in the submitted article.
